This article has been retracted.

# Analysis of the Effect of Fast Recovery Surgery Concept on Perioperative Nursing Care of Patients with Radical Resection of Cervical Cancer and Its Influence on Psychological Status

**DOI:** 10.1155/2022/2023159

**Published:** 2022-08-09

**Authors:** Yun Lu, Luxi Xu, Xiaoyu Lin, Xueling Qi, Ling Xia, Yuan Wang

**Affiliations:** ^1^Department of Obstetrics and Gynecology, Affiliated Hospital of Jiangnan University, Wuxi, China; ^2^Department of Pediatrics, Affiliated Hospital of Jiangnan University, Wuxi, China

## Abstract

**Objective:**

To explore the applied effect of fast-track surgery concept in the perioperative nursing of patients undergoing radical cervical cancer surgery and its influence on mental state.

**Methods:**

The clinical data of 110 patients undergoing radical cervical cancer surgery in our hospital from May 2015 to May 2017 were retrospectively analyzed, and they were randomly divided into a research group (*n* = 55) and a reference group (*n* = 55). The reference group received routine clinical nursing, and the research group received fast-track surgical nursing. Then, we compared their nursing effect and influence on the mental state of patients in the two groups.

**Results:**

The Karnofsky performance status (KPS) scores of patients in the two groups after intervention were significantly lower than those before the intervention (*P* < 0.001), and after intervention, patients in the research group had significantly lower KPS scores as compared to patients in the reference group (*P* < 0.001). There was a significant decrease in the self-rating anxiety scale (SAS) scores and self-rating depression scale (SDS) scores of patients in the two groups after intervention in comparison with before intervention (*P* < 0.001), and patients in the research group after intervention had significantly lower SAS and SDS scores compared to the reference group (*P* < 0.001). Patients in the research group spent short time on expelling gas, eating, and getting out of bed as compared to the reference group (*P* < 0.001); after intervention, compared to patients in the reference group, patients in the research group had significantly higher scores in cognitive function, emotional function, social function, and physical function (*P* < 0.05). There was no significant difference in IgA, IgM, and IgG levels before intervention (*P* > 0.05). After intervention, the IgA, IgM, and IgG levels of patients in the two groups were all lower than before intervention, and patients in the research group had significantly higher IgA, IgM, and IgG levels as compared to the reference group (*P* < 0.001); the complication rate of patients in the research group was significantly lower than that in the reference group (*P* < 0.05).

**Conclusion:**

The fast-track surgery concept effectively helps improve the negative emotion of patients, shorten recovery time, improve quality of life, and reduce the impact on immune function in the radical cervical cancer surgery, and it is worthy of promotion and application, with a high safety.

## 1. Introduction

Cervical cancer is a common gynecological malignant tumor, with insidious symptoms in the early stage and abnormal vaginal bleeding in the late stage. Therefore, regular physical examination and vaccination can effectively prevent and control the occurrence of cervical cancer [1]. The latest data released by the WHO [2] shows that there are about 570,000 patients with cervical cancer worldwide, with an increase of 2.3–3.4% by year, and a mortality of 54.29%. The Yellow Emperor's Classic of Internal Medicine attributed cervical cancer to the categories of “vaginal sore” and “qi deficiency.” Traditional medicine believes that the occurrence of this disease is mostly related to the internal injury of the emotions, eating disorders, early marriage, and unclean and multiple sexual intercourse. These factors act on the body, causing dysfunction of the liver, spleen, and kidneys, disharmony of qi and blood, damage to Chong and Ren, and missed pulses, leading to damp-heat, phlegm-dampness, and stasis toxin that invade the uterus. In addition to oral administration of medicines, the treatments also included vaginal administration, traditional Chinese medicine retention enema, traditional Chinese medicine injection, acupuncture, and other methods. According to the pathogenesis and etiology of traditional Chinese medicine, the treatment is mostly based on strengthening the righteousness and eliminating the pathogens to prolong the life of the patient.

More importantly, since the first licensed vaccine for prevention of morbidity and mortality attributable to human papillomavirus (HPV)-associated disease, it has presented the potential to eliminate cervical cancer less than 4 new cases per 100000 women years. HPV is one of the most common sexually transmitted infections and a well-established cause of cervical cancer, and the total burden of cervical cancers attributable to HPV is substantial.

At present, surgery is still an effective measure to treat cervical cancer. Radical cervical cancer surgery is suitable for patients in the early stages I-II, and its advantage is to help young patients preserve ovary and vaginal function [3, 4]. Despite the remarkable effectiveness, it is associated with complications such as urinary retention, anemia, intestinal obstruction, lower extremity edema, and ureteral leakage, resulting in the irritability and anxiety of patients after operation, affecting the prognosis. All these might be attributed to the fact that general surgery gives rise to a certain immunosuppressive effect on patients after surgery. With the continuous development of medical technology, the requirements for surgical treatment have increased as well. Therefore, it is particularly important to reduce the damage and improve the postoperative negative emotion on the basis of ensuring the treatment effect. Effective nursing plan is capable of improving the perioperative indexes of patients with cervical cancer, reducing the mental burden and clinical complications, and accelerating their recovery [5]. Fast-track surgery is a perioperative nursing concept that integrates multiple disciplines through continuous optimization of nursing procedures, the decrease in surgical trauma and the improvement of quality of life. In this study, the major objective was to analyze the impact of routine clinical nursing and fast-track surgical nursing on the perioperative period of patients undergoing radical cervical cancer surgery.

## 2. Materials and Methods

### 2.1. General Materials

The clinical data of 110 patients who underwent radical cervical cancer surgery in our hospital from May 2015 to May 2017 were retrospectively analyzed, and patients were randomly divided into a research group (*n* = 55) and a reference group (*n* = 55). The average age of patients in the research group was (47.52 ± 4.52) years old. According to the diagnostic criteria of TNM Classification of Malignant Tumors [6], the research group consisted of 19 patients at stage Ia and 36 patients at stage Ib, and they were 16 patients with squamous cell carcinoma, 21 patients with adenocarcinoma, and 18 patients with adenosquamous carcinoma in term of tumor type. In the reference group, there were 21 patients at stage Ia and 34 patients at stage Ib, with the average age of (47.49 ± 4.51) years old, and they were 14 patients with squamous cell carcinoma, 23 patients with adenocarcinoma and 18 patients with adenosquamous carcinoma in term of tumor type.

### 2.2. Inclusion Criteria

The inclusion criteria were as follows: patients who met the clinical diagnostic criteria of cervical cancer, patients who had clear awareness and could follow our instruction, patients aging 23–67 years old, and this study was approved by the ethics committee, and patients and their families signed an informed consent letter given that they had known the aim and procedure of this study.

### 2.3. Exclusion Criteria

The exclusion criteria were as follows: patients with other cancer, patients with coagulation dysfunction or systemic immune diseases, patients with palliative surgery, and patients with a history of pelvic surgery.

## 3. Methods

The reference group received routine perioperative nursing, and we formulated specific nursing plans based on the specific causes, conditions, and nursing results of patients, including clinical health education, medication guidance, hospitalization environment, and daily diet intervention. The research group received fast-track surgical nursing, and we made a personalized nursing plan on the basis of the specific condition of patients. This plan was drafted according to the Expert Consensus and Path Management Guide for Fast-track Surgery (2016version) [7], including the measures such as psychological counseling, preoperative preparation, intraoperative nursing, and postoperative recovery instruction, which minimized intraoperative risks and increased the success rate. Based on the consensus of experts, our department initially formulated the enhanced recovery nursing plan for radical cervical cancer, and the primary nurses checked if the above plan had been completely performed. Psychological counseling: we communicated with patients before operation, discovered their mental problems in time, and then patiently helped eliminate their inner tension and fear, so that patients followed the surgical treatment. Intestinal preparation: we instructed patients to fast for 6 hours before operation and drank 350 ml of 12.5% glucose at 2 hours before operation. Intraoperative nursing: we strictly controlled the infusion rate, kept patients warm, and then removed the abdominal drainage tube after operation. Postoperative nursing: patients were gradually back to a normal diet within 3-4 days after operation, and we encouraged patients to get out of bed, relax leg once every 20 minutes after operation, turn over once every 2 hours, and walk properly with the assistance of nurses after 6 hours of getting out of bed. On the first day after surgery, patients excised on your own and adjusted the amount of exercise appropriately. On the third day after surgery, nurses helped clamp the urinary tube and open it at regular intervals. On the 6^–^8th day after surgery, nurses removed the urinary tube and kept patients warm. In accordance with the postoperative recovery of patients, we made a specific discharge plan and informed them and their family members of the precautions after discharge.

### 3.1. Observation Indexes

Referring to the Karnofsky performance status (KPS) scale [8], the systemic symptoms and signs of patients in the two groups before and after intervention were assessed, with a full score of 10 points. The score was directly proportional to the severity of the systemic symptoms of patients.

Referring to the self-rating depression scale (SDS) [9] and self-rating anxiety scale (SAS) [10], the degree of depression and anxiety before and after intervention were evaluated, with a full score of 100 points for each scale. The degree of depression and anxiety was directly proportional to the scores.

The first time to expel gas, eating time, and time to get out of bed between the two groups were recorded.

The quality of life of patients in the two groups after intervention was evaluated according to the quality of life (QOL) for patients with cancer [11] including cognitive function, emotional function, social function, and physical function, with a full score of 100 for each factor. The score was directly proportional to the quality of life of patients.

3 ml of fasting venous blood of patients before and after intervention was collected, centrifuged to obtain serum, and immunoglobulin A (IgA), immunoglobulin M (IgM), and immunoglobulin G (IgG) were detected by the turbidimetric inhibition immunoassay.

Complications incidence of patients in the two groups were recorded and counted.

### 3.2. Statistical Methods

SPSS 20.0 software was used to statistically analyze and process all the data in this study. The enumeration data were expressed by (*n* (%)), using the *x*^2^ test, and the measurement data were expressed by (*x* ± *s*), using the *t*-test. *P* < 0.05 meant that the difference was statistically significant.

## 4. Results

### 4.1. Baseline Data

There was no significant difference in the baseline characteristics of patients in the two groups (*P* > 0.05), and they were comparable.

### 4.2. Comparison of KPS Scores before and after Intervention

The KPS scores of patients in the two groups after intervention were significantly lower than those before intervention (*P* < 0.001), and patients in the research group after intervention had significantly lower KPS scores as compared to patients in the reference group (*P* < 0.001), as shown in Figure 1.

### 4.3. Comparison of SAS and SDS Scores before and after Intervention

After intervention, the SAS and SDS scores of patients in the two groups were significantly lower than those before intervention (*P* < 0.05), and patients in the research group had significantly lower SAS and SDS scores as compared to patients in the reference group (*P* < 0.05), as given in Table 1.

### 4.4. Comparison of Various Recovery Indexes

Patients in the research group spent shorter time on first expelling gas, eating, and getting out of bed as compared to patients in the reference group (*P* < 0.001), as shown in Figure 2.

### 4.5. Comparison of QOL Scores after Intervention

The scores of cognitive function, emotional function, social function, and physical function of patients in the research group after intervention were significantly higher than those in the reference group (*P* < 0.001), as given in Table 2.

### 4.6. Comparison of Various Immune Indexes before and after Intervention

There was no significant difference in the levels of IgA, IgM, and IgG between the two groups before intervention (*P* > 0.05). After intervention, the levels of IgA, IgM, and IgG in the two groups all decreased, and patients in the research group had significantly higher levels of IgA, IgM, and IgG as compared to the reference group (*P* < 0.05), as given in Table 3.

### 4.7. Comparison of Postoperative Complications

Patients in the research group had significantly lower total incidence of complications compared to patients in the reference group (*P* < 0.05), as given in Table 4.

## 5. Discussion

In the early stage, the hidden symptoms of cervical cancer result in the continuous increase in prevalence and mortality. Surgical treatment plays a critical role in the treatment of cervical cancer, but the trauma caused by surgery remains an inescapable issue in the medical field [12]. Trauma reduces the immunity of patients, induces a variety of diseases, and then affects the prognosis. Some scholars believe that the application of effective clinical nursing pathways in the perioperative period of radical cervical cancer can greatly reduce the occurrence of trauma and postoperative complications and improve the quality of life [13]. The concept of fast-track surgery has been widely used in developed regions such as Europe and the United States and gradually accepted by Chinese doctors. This concept was first applied to gastrointestinal surgery, with remarkable results, and gradually applied to other types of surgery [14, 15].

This study found that after patients in the research group receiving the fast-track surgical nursing spent significantly shorter time on expelling gas, eating, and getting out of bed as compared to patients in the reference group, suggesting that this nursing plan is beneficial to the postoperative recovery of patients with cervical cancer. In the meantime, fast-track surgical nursing, a comprehensive nursing model that integrates multiple disciplines, emphasizes patient-centered care and formulates a specific nursing plan in the physical and psychological aspects according to their conditions to reduce negative emotion and improve their treatment confidence [16]. This study discovered that the SAS and SDS scores of patients in the research group after intervention were significantly lower than those in the reference group. Hoffman et al. [17] pointed out that fast-track surgical nursing were applied to the modified radical mastectomy for breast cancer, and the SAS score of patients after intervention was significantly lower than that of the control group (58.03 ± 3.16) vs. (64.13 ± 3.25), indicating that in the implementation of fast-track surgical nursing. This might be because we accurately acquired the mental state of patients through active communication with them and promptly helped them effectively relieve their depression, anxiety, and other negative emotions. Radical cervical cancer surgery damages the tissues of patients, resulting in the decrease in immunity after surgery. The function of the immune system is to defend against the invasion of external organisms including viruses and bacteria and suppress rebellious cells such as cancer cells. The immune system or cells mainly rely on innate immunity, specific immunity, and humoral immunity to kill or eliminate pathogens in the body [18].

Promisingly, in this study, it was confirmed that the IgA, IgM, and IgG levels of patients in the research group after intervention were significantly higher than those in the reference group, indicating that the implementation of fast-track surgical nursing reduced the damage and the impact on internal immune cells to improve surgical safety. Conversely, routine perioperative clinical nursing forbidding food and drink affected the intestinal function of patients, which resulted in imbalance of gut flora and an increase in the probability of complications, and also caused electrolyte disorders in the body and affecting the prognosis [19]. This study confirmed that the concept of fast-track surgery, a reliable clinical nursing measure, reduced the incidence of postoperative complications in patients. The limitations of this study were small size samples, lack of the long-term prognosis, and the influence of subjective factors in the implementation of nursing plan.

In conclusion, fast-track surgical nursing intervention improves the negative emotion of patients, speeds up their recovery, and reduces damage to the immune cells, with good safety and efficacy profiles. It is worthy of promotion and application.

## Figures and Tables

**Figure 1:** Comparison of KPS scores before and after intervention (*x* ± *s*, scores). The *X*-axis indicates before and after intervention, and the *Y*-axis indicates KPS (scores). The KPS scores of patients in the research group before and after intervention were (5.84 ± 0.56) and (3.12 ± 0.37), respectively. The KPS scores of patients in the reference group before and after intervention were (5.81 ± 0.54) and (4.39 ± 0.43), respectively. ^*∗*^Significant difference in the KPS scores of the research group before and after intervention (*t* = 30.054, *P* < 0.001). ^*∗∗*^KPS scores of the reference group before and after intervention are significantly different (*t* = 15.256, *P < *0.001). ^*∗∗∗*^KPS scores of patients in the two groups after intervention are significantly different *(t = *16.603, *P* < 0.001).

**Figure 2:** Comparison of various recovery indexes after operation (*x* ± *s*). The *X*-axis represents the first time to expel gas, eating time, and the time to get out of bed, and the *Y*-axis represents the recovery time, h. The first time to expel gas, eating time, and time to get out of bed in the research group were (20.58 ± 3.44) h, (7.26 ± 1.64) h, and (19.87 ± 3.88) h, respectively, and the first flatulence time, eating time, and time to get out of bed in the reference group were (37.23 ± 3.51) h, (9.41 ± 1.57) h, and (24.46 ± 3.74) h, respectively. ^*∗*^Significant difference in the first time to expel gas between the two groups (*t* = 25.125, *P* < 0.001). ^*∗∗*^Significant difference in the eating time between the two groups (*t* = 7.023, *P* < 0.001). ^*∗∗∗*^Significant difference in the time to get out of bed between the two groups (*t* = 6.317, *P* < 0.001).

**Table 1:** Comparison of SAS and SDS scores before and after intervention (*x* ± *s*, scores).

Indexes	Time	Research group (*n* = 55)	Reference group (*n* = 55)
SAS scores	Before intervention	67.25 ± 5.63	67.28 ± 5.59
	After intervention	57.36 ± 3.21	63.75 ± 3.52^*∗*^

SDS scores	Before intervention	66.42 ± 3.47	66.39 ± 3.52
	After intervention	56.31 ± 4.26	62.19 ± 3.48^*∗*^

The SAS and SDS scores of patients in the two groups after intervention were significantly lower than those before intervention. ^*∗*^Comparison of the research group and the reference group after intervention (*P* < 0.05).

**Table 2:** Comparison of QOL scores after intervention (*x* ± *s*, scores).

Group	*n*	Cognitive function	Emotional function	Social function	Physical function
Research group	55	51.69 ± 8.35	64.02 ± 7.44	40.17 ± 7.67	31.56 ± 6.85
Reference group	55	47.23 ± 8.17	55.28 ± 7.36	33.56 ± 7.73	22.69 ± 6.74
*t*		2.831	6.194	4.502	6.845
*P*		0.006	<0.001	<0.001	<0.001

**Table 3:** Comparison of various immune indexes before and after intervention (*x* ± *s*, g/L).

Indexes	Time	Research group (*n* = 55)	Reference group (*n* = 55)
IgA	Before intervention	2.57 ± 0.38	2.54 ± 0.41
	After intervention	2.42 ± 0.32^*∗*^	1.94 ± 0.28

IgM	Before intervention	1.91 ± 0.26	1.88 ± 0.27
	After intervention	1.64 ± 0.34^*∗*^	1.32 ± 0.22

IgG	Before intervention	10.59 ± 2.13	10.61 ± 2.15
	After intervention	9.85 ± 2.02^*∗*^	8.04 ± 2.26

^*∗*^Comparison with the reference group after intervention (*P* < 0.05).

**Table 4:** Comparison of postoperative complications (*n* (%)).

Group	*n*	Infection	Urinary retention	Pain	Total incidence
Research group	55	1 (1.82%)	0 (0.00%)	2 (3.64%)	5.45% (3/55)
Reference group	55	4 (7.27%)	2 (3.64%)	4 (7.27%)	18.18% (10/55)
*X* ^2^					4.274
*P*					0.039

## Data Availability

No data were used to support this study.
